# The taoist culture and the digital economy: Evidence from Chinese cities

**DOI:** 10.1016/j.heliyon.2023.e22846

**Published:** 2023-12-01

**Authors:** Xiaohui Chen, Xing Wu

**Affiliations:** a School of Digital Economics, Sichuan University Jinjiang College, Meishan, China; b Chengdu Technological University, School of Economics & Management, Chengdu, China

**Keywords:** Taoist culture, *Tao Te ching*, Digital economy

## Abstract

A key component of China's national plan is now the growth of the digital economy. This development relies on the continuous and in-depth practice of the vast majority of Chinese people who are deeply influenced by Chinese culture, of which Taoist culture is an important component that is closely related to the Chinese people and deeply influences overall worldviews. How does Taoist culture affect digital economy growth? Applying a theoretical analysis, in order to investigate this subject, this study used a two-way city–year fixed effects model with Chinese city data. The results demonstrate that Taoist culture can promote digital economy growth. The reason for this is that the “action” of Taoist culture refers to doing what should be done rather than inactivity. Additionally, the “quietness” of Taoist culture facilitates public individuals' single mindedness. The findings imply that Taoist culture has financial decentralization and financial technology effects. Theoretically, improvement in the degree of financial decentralization and technology can promote cities' digital economy development.

## 1 Introduction

Taoist culture is one of the main pillars of traditional Chinese culture [1] that is closely related to general public sentiment [2] and alleviates spiritual pressure and addresses the spiritual needs of the Chinese people [3]. The imagination and creativity of the adventurous concept of “immortality never dies” in Taoist culture is similar to Western science (speculative) fiction perspectives, influencing contemporary Chinese people to activate their thinking, stimulate imagination, innovate, and advance great achievements in innovation [4]. Developed and developing countries prioritize digital economy development, which has been elevated as an integral aspect of China's national strategy. Industrial digitization and digital industrialization are the two main facets of the digital economy, both of which are inseparable from the Chinese people's implementation of digital economy innovation. Taoist cultural proclivities can stimulate the imagination and creativity of Chinese people [4]. China is one of the world leaders in the growth of its digital economy. **Does China's highly developed digital economy stem from Taoist culture?** In order to highlight China's cultural experience in promoting the growth of the digital economy in developing nations worldwide, this study investigates the effects and workings of Taoist culture on the digital economy.

Digital technology businesses in domains including artificial intelligence, blockchain, cloud computing, big data, and the Internet of Things—collectively known as ABCDI—are essential to the development of the digital economy. These digital technologies began large-scale commercial application in the early 21st century, and enterprises in first, second, and third industries three industrial began to apply digital technologies to production and business activities to improve efficiency, increase output, and gain competitiveness in implementing emerging innovations and benefiting nondigital technology enterprises in the three industries. In short, digital economy development is inseparable from digital innovation. As an important component of Chinese culture, Taoist culture has a long history and profound societal influence [5]. As a native faith in China, Taoist culture is closely related to traditional beliefs and is often considered to be an important force that influences Chinese beliefs [3] that can stimulate the Chinese imagination and creativity [4]. Therefore, **we hypothesize that Taoist ideology can promote digital economy development.** Notably, digital economy development cannot progress without financial support. The basic concept of Taoist culture is “tranquility” [6,7], which can inspire people to think calmly and inspire inspiration [8]. The Taoist ideology of “the ruler does nothing but the minister does something” motivates Chinese people not to act recklessly, to operate according to existing rules, and to streamline administration and delegate power [7]. These concepts are conducive to improving local governments' promotion of financial decentralization, growth of digital economies and financial technologies. Therefore, **we hypothesize that Taoist culture promotes the growth of the digital economy in China by improving local governments’ financial decentralization and financial technology innovation efforts**.

**Our study adds to the body of knowledge about the beneficial effects of China's indigenous Taoist culture.** Existing literature has studied the influence of Taoist culture from macro [9,10] and micro [[11], [12], [13]] perspectives. From a macro perspective, Chen et al. (2023) found that Taoist culture encourages the growth of digital inclusive finance, showing that a city's level of development of digital inclusive finance will increase with the strength of its Taoist culture [9]. Taoist culture has been found to enhance tourists' loyalty to Taoist tourism products, which promotes tourism industry development [10]. At the micro level, Shao et al. (2023) determined companies in areas with strong Taoist culture to be more charitable but invest less in the environment [11]. Taoist culture instills respect and love for life, which can improve individuals' social qualities [13] and enhance Chinese enterprises' management [12]. In addition, Taoist culture advances low-carbon practices among employees [14]. Overall, extensive research has been conducted regarding the positive impact of Taoist culture; however, seldom has the connection between Taoist culture and the digital economy been discussed. Our research enriches previous research on the positive impact of Taoist culture.

**This study adds to the body of knowledge already available on the digital economy.** Previous research has looked at how the digital economy is affecting the economy [[15], [16], [17], [18]] and its influencing factors [[19], [20], [21], [22]] extensively. With regards to the economic implications, the digital economy stimulates enterprises' transition to renewable energy by enhancing governance capabilities [17], which reduces carbon dioxide emissions [15,16]. The digital economy plays a crucial role in facilitating regional low-carbon development and in supporting China's pursuit of high-quality economic growth [18]. Regarding influencing factors, novel development, massive market scale, institutional constraints, the legal system, and tax policies related to prevention and control of the COVID-19 pandemic affected digital economy development [20,21]. The utilization of digital technology, particularly artificial intelligence, plays a pivotal role in the progression of the digital economy [19]. Furthermore, the stimulation of technological innovation through financial technology contributes to the advancement of China's provincial-level digital economy [22]. Overall, previous studies have extensively investigated the factors that influence the development of the digital economy; however, investigations of the influencing factors of digital economy development from a cultural perspective are minimal. This study investigates the factors that influence the development of the digital economy from a research perspective.

The subsequent sections of this work are organized in the following manner. In second section, we give a comprehensive theoretical analysis. Section 3 elucidates the research strategy, section 4 scrutinizes the outcomes of the empirical analysis, and section 5 performs associated mechanism tests while summarizing the findings.

## 2 Theoretical analysis

### 2.1 Impact analysis

Since 2008, the profound incorporation of ABCDI digital technologies within the global economy has effectively contributed to the establishment of the digital economy [22]. The digital economy encompasses the processes of digital industrialization and industrial digitization [23], both of which require enterprises to implement and advance innovation. **First**, regarding enterprise innovation, previous studies have found that stimulating employees' creativity is the key to promoting employee innovation practices [24]. Creative employees prefer to engage in risky, uncertain, and challenging work [25], which can advance enterprises' innovation. This means that employees' creativity must be stimulated to promote enterprise innovation. **Second**, previous studies have determined guidance related to creativity and innovation, supporting employees' independent pursuit of new ideas, and respecting individuality is beneficial for promoting innovation practices [26,27]. This requires managers to become less conservative, traditional, and paternalistic [25] and actively release controlling behaviors. **Third**, previous research has suggested that motivating employees’ work engagement will stimulate them to invest more time and energy toward work, become more focused and hardworking, and enhance the ability to withstand failures and setbacks. Such employees are courageous enough to accept challenges, actively seek solutions, and strive to overcome various difficulties encountered in their work [28], overcoming the many challenges faced by enterprises in innovation, which advances enterprise innovation.

Taoist culture is an important component of Chinese culture [5,29] that is embedded in Chinese society [2] and deeply influences managers of Chinese enterprises, which can advance digital economy development. **First**, Taoist culture stimulates Chinese people to pursue digital innovation. The imagination and creativity of novel ideas inherent to Taoist culture has a similar influence as Western science (speculative) fiction thinking, and helps Chinese people to activate their creativity, stimulates the imagination, breaks through the old and introduces new approaches, and facilitates achievements in digital innovation [4]. **Second**, Taoist culture enables Chinese people to delegate independent tasks to subordinates to advance digital innovation. The concept of “inaction” in Taoist culture, indicating that “the king does nothing but the minister does something” has been adopted by management scientists worldwide [30]. This inaction requires individuals to avoid acting recklessly but to follow the law [7]. Enterprise managers who are familiar with Taoist culture do something but do nothing in implementing management policies. In digital innovation, enterprise managers who embrace Taoist culture will courageously delegate power and allow employees to boldly implement independent digital innovation, ultimately advancing digital economy development. **Third**, Taoist culture spurs Chinese people to focus on digital innovation. “Quietness” is another basic concept of Taoist culture, and its pursuit can nurture a calm demeanor [6,7], stimulate inspiration, and encourage individuals to immerse themselves into innovation [8]. Therefore, management approaches that are informed by Taoist culture can motivate people to engage in digital innovation, advancing digital economy development.

In essence, the cultural principles of Taoism create an environment that supports managers in their efforts to encourage, delegate, and prioritize digital innovation, hence promoting the development of the digital economy. Thus, this study posits the subsequent hypothesis.

H1 Taoist culture promotes digital economy development.

### 2.2 Mechanism analyses

The advancement of the digital economy necessitates the integration of digital technical innovation inside digital technology firms, as well as the adoption of digital transformation and innovation by non-digital technology enterprises, both of which are inseparable from finance. This study aims to examine the effects of financial decentralization and financial technology on many aspects of the finance sector.

#### 2.2.1 Financial decentralization channels

In order to expedite China's economic transition, the central government has opted to partially devolve its control and decision-making authority pertaining to the allocation of financial resources to local governments (i.e., city governments), establishing financial decentralization for local governments [22]. Under this institutional framework, determining the actual amount of financial decentralization obtained by local governments depends on many factors.

**Taoist culture can improve cities' degree of financial decentralization via the following mechanisms**. **First**, financial risks are controlled. The basic concept of quietness in Taoist culture pursues spiritual specificity [6,7], causing people to think calmly and inspiring innovation [8], which encourages local financial regulatory institutions to control the financial risks associated with financial decentralization in a focused and calm manner, improves risk control capabilities, and encourages local governments to courageously pursue financial decentralization. **Second**, financial decentralization innovation is authorized. The inaction perspective of Taoist culture can inspire local governments to govern following the Tao, not act recklessly, and follow the law [7], while also simplifying administration and delegating power [7]. This encourages local financial organizations directly under local governments' jurisdiction to actively implement financial product innovation to improve competitiveness for financial resources and enhance financial decentralization. **Third**, innovation in financial decentralization is encouraged. Taoist culture motivates Chinese people to activate creative thinking, stimulate their imaginations, and produce new approaches [4]. The Tao can accelerate people's awareness and innovation, which advances local governments' promotion of financial decentralization innovation and raises financial decentralization levels.

**The advancement of the digital economy is facilitated by the level of financial decentralization in cities, which can be attributed to the following processes. First** crucial aspect to consider is the significance of financial assistance. Improving a city's financial decentralization can expand the availability of debt financing for local enterprises, providing the necessary financial support to implement digital innovation and promote local digital economy development. **Second** is the role of risk taking. Based on financial decentralization, local governments can be financed through local financial organizations to support the development of innovative enterprises. Therefore, financial decentralization improves the degree of regional innovation [31], which improves enterprises' risk taking practices [32], encouraging risk taking activities related to digital innovation, and promoting digital economy development. **Third**, due diligence also has a promotional role. In addition to providing financial support, financial decentralization can improve the availability of debt financing for local enterprises and promote enterprise managers' due diligence, which encourages enterprise managers to actively promote digital innovation to improve total factor productivity, supporting local digital economy growth.

In summary, Taoist culture can improve cities’ degree of financial decentralization and promote digital economy growth. Consequently, the present investigation posits the subsequent hypothese.

H2 Taoist culture promotes digital economy development by improving cities' degree of financial decentralization.

#### 2.2.2 Financial technology channels

Since the onset of the 21st century, financial businesses have progressively enhanced the incorporation of digital technologies, such as ABCDI, into their operational processes. This integration has facilitated the provision of financial services that are founded on digital technologies, thus giving rise to the emergence of financial technology (fintech) [22,23]. Financial technology has multiple benefits, and countries around the world have been vigorously promoting its development. Similarly, the development of fintech is influenced by many factors.

**Taoist culture can improve cities' degree of fintech**. **First**, financial risks are controlled. Taoist culture, which takes quietness as one of the basic concepts, pursues spiritual specificity [6,7], causing people to think carefully and inspiring innovation [8]. This causes financial enterprises to navigate financial technology risks in a single minded and calm manner, and encourages financial enterprises to courageously conduct financial technology innovation and improve cities' degree of level financial technology. **Second**, financial technology innovation requires financial enterprises' boards of directors to delegate power and fearlessly eliminate direct constraints. Similarly, the Taoist concept of inaction can constrain financial enterprises' boards from reckless practices, encouraging the delegation of power to enterprise managers [7] to promote financial technology innovation and finally improve the degree of financial technology. **Third**, Taoist precepts stimulate financial innovation. Financial technology innovations are unprecedented and disruptive, requiring considerable imagination and creativity. The promotion of imagination and creativity via fantastic ideas in Taoist culture motivates Chinese people to activate creative thinking, stimulate their imaginations, and produce novel innovations [4], which actively promote financial enterprises’ financial technology innovation.

**Cities' degree of financial technology advances digital economy development**. **First**, it introduces positive incentives. To meet banks' need for risk assessment using financial technology and expanded credit support, enterprises are compelled to promote digitization. Therefore, financial technology has a positive incentivizing influence on enterprises' digitization and promotes digital economy development. **Second** is the role of financial support. High-quality financial services can provide expanded financial support for enterprises' digital transformation [33] to promote digital economy development. **Third** is fintech's leading role. The advancement of financial technology fosters the progress of information and communications technology in the region, driven by market demand, hence promoting the growth of digital industrialization. In addition, the field of financial technology plays a crucial role in creating a conducive information technology infrastructure that enables businesses to effectively undertake digital transformation and innovation. This, in turn, facilitates the advancement of industrial digitalization and contributes significantly to the growth of the digital economy.

In summary, fundamental aspects of Taoist culture can improve cities’ degree of financial technology to promote digital economy development. Consequently, the present investigation posits the subsequent hypothesis.

H3 Taoist culture promotes digital economy development by improving cities' degree of financial technology.

## 3 Materials and methods

We follow the mainstream research methods of contemporary economics, conducting the above theoretical analysis and proposing three hypotheses, followed by empirical testing. The following research design is conducted.

### 3.1 Data

Conducting research at the city level is the first choice for scholars when investigating Chinese issues (e.g., Chen et al., 2023) [9]. We use all cities in China as our sample, obtaining data from 229 cities after excluding missing data. This study references Yin and Peng (2020) [34], using the Digital Inclusive Finance Index developed by Peking University, which began collecting relevant data in 2011, as the proxy variable for fintech. The China City Statistical Yearbook serves as the source for acquiring additional city data. After 2019, the *Yearbook* ceased disclosing data on foreign direct investment, which is a crucial variable for our empirical research. Therefore, empirical testing was conducted using data collected from 229 cities in China over the period spanning between 2011 and 2019.

Referencing optimized calculation schemes from Liang et al. (2021) [35], this study aims to assess the level of digital economy development at the city level by obtaining the regional digital economy development index. The digital economy development index for cities is calculated for the years 2011–2019. In order to assess the prevalence of Taoist culture in various cities, we conducted an analysis by referring to the data provided by the State Administration of Religious Affairs. By identifying and documenting the locations where Daoist temple is, we were able to estimate the extent of Taoist cultural influence in each respective city.

The quantity of patent applications pertaining to digital technologies (i.e., ABCDI) required for determining cities' digital economy development index are obtained from the Patsnap website (patsnap.com). The word frequency of relevant keywords is obtained from the People's Daily Online referencing Chen and Zhang (2021) [32]. Each city's carbon emissions are obtained from the China Emission Accounts and Datasets, and additional statistics are acquired from the People's Bank of China, National Bureau of Statistics of China, the Ministry of Civil Affairs of China, and the WIND database. Continuous variables are winsorized by 1 % to eliminate the influence of outliers.

### 3.2 Models

#### 3.2.1 Model of H1

Due to the static nature of the number of Taoist temples across time, it is not feasible to test hypothesis H1 with city fixed effects. Referencing Chen et al. (2023) [9], the design of the model involves the use of a two-way fixed effects time-province:

(1) $$Deco_{it}=\alpha_{0}+\beta_{1}*DJ_{i}+\eta *X+\alpha_{t}+\lambda_{ik}+\varepsilon_{it}$$

where $Deco_{it}$ represents the digital economic development index of city *i* in year *t*, $\alpha_{0}$ is the constant term, $\alpha_{t}$ is the year fixed effect, the variable $\lambda_{ik}$ represents the fixed effect of the k-th province in which city *i* is situated. and $\varepsilon_{it}$ is the randomized perturbation term. $DJ_{i}$ represents the independent variable, indicating Taoist culture intensity in city *i* and $\beta_{1}$ is its coefficient. When $\beta_{1}$ is significantly positive, this indicates that Taoist culture promotes digital economy development. The control variable, denoted as *X*, is defined and explained in the following manner.

#### 3.2.2 H2 and H3 models

To test the H2 and H3 research hypotheses, The models (2)-(4) aim to examine the impact processes discussed above, drawing upon the works of Wen and Ye (2014) [36] and Chen et al. (2023) [9] for reference.

(2) $$Deco_{it}=\alpha_{0}+\beta_{1}*DJ_{i}+\eta *X+\alpha_{t}+\lambda_{ik}+\varepsilon_{it}$$

(3) $$med_{it}=\alpha_{0}+\xi *DJ_{i}+l*X_{1}+\alpha_{t}+\lambda_{ik}+\varepsilon_{it}$$

(4) $$Deco_{it}=\alpha_{0}+\beta_{1}*DJ_{i}+\delta *med_{it}+\eta *X+\alpha_{t}+\lambda_{ik}+\varepsilon_{it}$$

The variable $med_{it}$ represents the mediating role of the city's degree of financial decentralization (*Fd*) and financial technology (*Fintech*). Initially, Equation (2) is estimated without the inclusion of any mediating variables. If the coefficient $DJ_{i}$, which represents the intensity of Taoist culture ($\beta_{1}$), demonstrates statistical significance, it suggests that Taoist culture has a comprehensive impact on the development of the digital economy. In such cases, further analyses can be pursued. Conversely, if the coefficient is not significant, it implies the presence of a masking effect. Furthermore, Equation (3) is employed to ascertain the impact of Taoist culture on the mediating factors. Next, we proceed to estimate Equation (4) following the inclusion of the mediating variable. If the coefficients ξ in Equation (3) and the coefficient δ in Equation (4) exhibit statistical significance, it suggests the presence of a mediating influence. If the coefficient $\beta_{1}$ in Equation (4) is statistically significant, it suggests that med_it has a partial mediating effect. If the observed result lacks statistical significance, it suggests that $med_{it}$ exhibits a complete mediating effect. In addition, when either the variable ξ in Equation (3) or the variable δ in Equation (4) demonstrates statistical significance, it is necessary to assess the mediating effect through the application of the Sobel test.

The control variable, denoted as *X* in Equations (2), (4), is consistent with the control variable in Equation (1). The control variable, denoted as $X_{1}$ in Equation (3), exhibits variability in accordance with the mediating variable. Below, we present additional information.

#### 3.2.3 Variables

The independent, mediating, and control variables are designed referencing the previous research, as shown in Table 1.

**Table 1:** Variable description.

	Variable	Symbol	Variable definition	References
Dependent variable	Digital economy development index	*Deco*	City digital economy development index calculated according to 7 indicators.	Liang et al. (2021), Zhao et al. (2020)
		*fDeco*	City digital economy development index calculated according to six indicators after excluding fintech	
Independent variables	Taoist culture intensity	*DJ*	Increase the count of Taoist temples in city by one unit and compute the natural logarithm of this value.	New in this article
		*rDJ*	The natural logarithm is derived by multiplying the quantity of Taoist temples in the city by the continuous time, incremented by one.	Yan and Lin (2019)
		*rrDJ*	The quantity of Taoist temples in a city is multiplied by the population density of the city and thereafter multiplied by the continuous variable of time.	Asc (1955)
Control variables	Population density	*Pden*	Total city population/land area	Arcand et al. (2015), Beck et al. (2000)
	Population growth rate	*Gpop*	Total city population increment/population of the previous year	
	Urbanization rate	*Rcity*	Urban population/total city population	
		*Rcity2*	*Quadratic term of Rcity*	
	Economic development level	*Lnpgdp*	Natural logarithm of city per capita real GDP	
	Financial development level	*Fsize*	City loan balance/GDP	
	Economic opening level	*Open*	City FDI/GDP	
	Industrial structure level	*Indstr*	1 * proportion of city primary industry + 2 * proportion of city secondary industry + 3 * proportion of city tertiary industry	
	Human capital level	*Hcap*	Number of city college students divided by total population	
	Financial autonomy	*Fiscal*	City fiscal revenue/City Fiscal Expenditure	
Intermediary variables	Financial decentralization level	*Fd*	City loan balance/national loan balance	He and Miao (2016)
	Financial technology level	*FinTech*	Beijing University Digital Inclusive Finance Index/100	Yin and Peng (2020)

##### 3.2.3.1 The dependent variable

The focal variable of this study pertains to the extent of advancement in the digital economy (*Deco*). Liang et al. (2021) [35] constructed the digital economy development index at the city level using five indicators. The digital economy is propelled by not only the internet but also by digital technologies such as ABCDI. Hence, this study uses the quantity of patent applications from cities as a proxy for measuring the extent of innovation in digital technology. Additionally, a word frequency analysis of 20 specific terms is utilized to gauge the level of enthusiasm exhibited by cities towards digital technology innovation. The present study formulates the digital economy development index by utilizing a set of optimal variables. The calculation of cities' digital economy development index (*Deco*) from 2011 to 2019 involves the utilization of factor analysis, with reference to the seven variables presented in Table 2.

**Table 2:** Index system of city digital economy development index.

Primary index	Secondary index	Original index	Reference
City digital economy development index	Internet consumer groups	Number of Internet users	Liang et al. (2021), Zhao et al. (2020)
	Internet-related practitioners	Number of computer service and software employees	
	Internet-related output	Telecom business volume	
	Mobile Internet consumption volume	Number of mobile phone users	
	Financial technology development	Peking University Digital inclusive financial index	
	ABCDI innovation enthusiasm	Word frequency of 20 keywords such as artificial intelligence, blockchain, cloud computing, big data and Internet of things.	Chen and Zhang (2021)
	ABCDI innovation output	Number of applications for five digital technology patents, including ABCDI	

Note: The keywords are the same as those used by Chen and Zhang (2021).

##### 3.2.3.2 Independent variable

The independent variable in this study is Taoist culture intensity (*DJ*). Taoist culture touches all aspects of traditional Chinese culture, and a contemporary phenomenon of advocating Taoist culture is occurring throughout China [29]. Taoist faith activity sites are permanent spaces for imparting Taoist ideas and conducting related activities. Such spaces are the carriers of Taoist culture and the window exposing the precepts of Taoist culture [3]. Hence, this study used the quantification of Taoist temples in each city as a proxy for measuring the degree of Taoist cultural presence. The variable *DJ* is derived by incrementing the count of cities' Taoist temples by one and thereafter applying the natural logarithm as a representative measure of Taoist cultural intensity.

In recent years, there has been a resurgence in the importance of traditional Chinese culture, coinciding with the development of the contemporary Chinese society and economy [37]. Consequently, the influence of Taoist culture is expected to rise over time. To control cities' individual fixed effects for the robustness check, referencing Yan and Lin (2019) [38], the number of Taoist temples in each city is multiplied as a continuous time variable, and the resulting value is transformed using the natural logarithm to yield *rDJ*. In addition, conformity (the phenomenon in which individuals maintain behavior that is consistent with collective opinions under the influence of groups) is a common social phenomenon that may also affect people's respect for Taoist culture. Herd behavior rises with the expansion of group size [39]. Hence, this study employs the product of the quantity of Taoist sites in each city, the city's population density, and the continuous time variable to derive *rrDJ* for the purpose of conducting a robustness analysis, in which a greater *DJ*, *rDJ*, and *rrDJ* indicates stronger Taoist culture intensity.

##### 3.2.3.1 Mediating variables

The variables that serve as mediators in this study are the extent of financial decentralization within cities and the utilization of financial technology

(1) Cities' degree of financial decentralization (*Fd*). Referencing He and Miao (2016) [40], the city loan balance/national loan balance represents the city's degree of financial decentralization.
(2) Cities' degree of financial technology (*Fintech*). Referencing Yin and Peng (2020) [34], the digital inclusive financial index characterizes cities' degree of financial technology.

The relationship between dependent variables, independent variables, mediating variables, and our hypotheses is illustrated in Fig. 1.

**Fig. 1:** Relationship between main variables and hypotheses.

##### 3.2.3.4 Control variables

For the control variables in Equation (1), this study constructs control variables such as population density, population growth rate, urbanization rate and its quadratic term, economic development level, financial development level, economic opening level, industrial structure level, human capital level, and financial autonomy referencing Chen et al. (2020) [41] and the existing economic development literature [42,43].

For the control variables in Equation (3), taking the degree of cities' financial decentralization as the dependent variable and referencing the existing literature, this study uses control variables of economic and financial development, regional opening level, urbanization rate, financial efficiency, fiscal policy, and government intervention. Taking cities’ degree of financial technology as the dependent variable, drawing upon the pertinent scholarly literature pertaining to technology innovation and financial innovation, this study uses the control variables of economic and financial development; regional opening, industrial structure, and human capital levels; urbanization rate, fiscal policy, government intervention, and financial efficiency.

## 4 Results

### 4.1 Descriptive statistics

Table 3 presents descriptive statistics for the main variables, revealing that the average city digital economy development index (*Deco*) is 4.0036, the minimum is 3.3196, the maximum is 7.2342. This indicates that cities' degree of digital economy development differs significantly, which aligns with the fundamental characteristics of uneven development across the nation. Fig. 2 illustrates the average and growth rate of China's urban digital economy development index from 2011 to 2019, revealing that the average urban digital economy development index in China increased from 3.4524 to 4.3852 in this period, with a compound annual growth rate of 3.03, which decreased from 8.38 % to 1.69 %. Second, the mean *DJ* value in cities characterized by a significant presence of Taoist culture is 2.5254, ranging from a low of 0.6931 to a maximum of 5.6454. These findings align with the broader national context of uneven development. Third, the mediating variables of financial decentralization and city financial technology development are also in accordance with the fundamental characteristics of uneven growth within the nation.

**Table 3:** Descriptive statistics of main variables.

Variable	Obs	Mean	Std. Dev.	Min	Max
*Deco*	1840	4.0036	0.5818	3.3196	7.2342
*DJ*	1840	2.5254	1.3060	0.6931	5.6454
*Fd*	1840	0.0327	0.0538	0.0013	0.5463
*FinTech*	1840	1.6374	0.6608	0.2948	2.8197
*Pden*	1840	0.4668	0.3202	0.0051	2.6483
*Gpop*	1840	0.0565	0.0512	−0.0692	0.2140
*Rcity*	1840	0.3465	0.2238	0.0468	1.0000
*Lnpgdp*	1840	1.4876	0.6522	−0.3594	3.5325
*Open*	1840	0.0186	0.0174	0.0000	0.1978
*Indstr*	1840	0.0236	0.0287	0.0183	1.2526
*Fsize*	1840	0.0966	0.0591	0.0114	0.7450
*Fiscal*	1840	0.5013	0.2319	0.0702	2.6651

**Fig. 2:** Average and growth rate of Chinese cities' digital economy development index (2011–2019).

Second, the mean Taoist cultural intensity *DJ* is 2.5254, with a minimum value of 0.6931 and a maximum value of 5.6454. These findings align with the prevailing national circumstances characterized by uneven development. This indicates that China's vast territory exhibits significant differences in Taoist culture intensity among cities, which align with the significant differences in the digital economy development index between cities. This also necessitates our further exploration of the impact of Taoist culture on digital economy development. Third, the mediating variables of cities' financial decentralization and financial technology development levels are consistent with the basic national conditions of unbalanced development.

### 4.2 Benchmark regression

The utilization of a double cluster adjustment technique for standard errors in both individual and time dimensions has the potential to mitigate the impact of autocorrelation and heteroskedasticity on the validity of statistical inference. By employing a gradual introduction of control variables, while controlling for time and province fixed effects, and utilizing robust standard error with dual individual and temporal clustering, we have estimated Equation (1). The findings of this estimation are displayed in Table 4.

**Table 4:** Regression results of equation (1).

	(1)	(2)	(3)	(4)	(5)
Variables	*Deco*	*Deco*	*Deco*	*Deco*	*Deco*
					
*DJ*	0.0646***	0.1026***	0.1047***	0.1022***	0.1014***
	(0.0222)	(0.0162)	(0.0161)	(0.0159)	(0.0158)
*Pden*		0.1910*	0.1759	0.1734	0.1678
		(0.1126)	(0.1097)	(0.1089)	(0.1085)
*Gpop*		0.3523***	0.3727***	0.3816***	0.3660***
		(0.1189)	(0.1189)	(0.1185)	(0.1186)
*Rcity*		−1.2383***	−1.3423***	−1.3472***	−1.3480***
		(0.2257)	(0.2149)	(0.2145)	(0.2146)
*Rcity2*		2.2341***	2.2484***	2.2310***	2.2319***
		(0.3087)	(0.3117)	(0.3116)	(0.3116)
*Hcap*		1.0858	0.8032	0.6892	0.6562
		(1.0500)	(1.0425)	(1.0274)	(1.0314)
*Lnpgdp*			0.1130***	0.1155***	0.0984**
			(0.0392)	(0.0393)	(0.0414)
*Open*			0.0359	0.0960	0.0309
			(0.4384)	(0.4419)	(0.4390)
*Indstr*			−0.3017***	−0.2937***	−0.3009***
			(0.0943)	(0.0923)	(0.0927)
*Fsize*				0.3712**	0.3745**
				(0.1704)	(0.1707)
*Fiscal*					0.0740
					(0.0510)
*Constant*	0.0646***	0.1026***	0.1047***	0.1022***	0.1014***
	(0.0222)	(0.0162)	(0.0161)	(0.0159)	(0.0158)
					
Individual	YES	YES	YES	YES	YES
Province	YES	YES	YES	YES	YES
					
Observations	1840	1840	1840	1840	1840
N	229	229	229	229	229
R^2^	0.5058	0.6429	0.6610	0.6711	0.6731

Robust standard errors are in parentheses; ***p < 0.01, **p < 0.05, *p < 0.1.

Columns (1)–(5) of Table 4 show that the *DJ* coefficients of Taoist culture intensity are significantly positive at the 1 % significance level, indicating that digital economy development can be improved by increasing Taoist culture intensity. The regression findings obtained from the benchmark analysis provide support for Hypothesis 1.

### 4.3 Robustness tests

In Columns (1)–(5) of Table 4, the coefficients of the independent variables are significant at the 1 % level, which can be considered a robustness check. This study also conducts further robustness tests through endogeneity treatment, replacing dependent variables, replacing independent variables, changing estimation model, and adding control variables.

#### 4.3.1 Endogeneity treatment

The empirical results demonstrate that Taoist culture can promote digital economy development. In contrast, as an important aspect of Chinese culture, Taoist faith has an extensive history [5], and the contemporary digital economy originated in 2008, making it challenging for the digital economy to affect Taoist culture. Nevertheless, it is important to acknowledge that the degree of Taoist culture (*DJ*) could potentially be endogenous due to the presence of measurement errors or unobservable factors. This analysis incorporates the findings of Kim et al. (2014) [44] and Chen et al. (2023) [9], utilizing the average Taoist cultural intensity in comparable cities during the identical year as the instrumental variable (IV) *ivDJ*. The influence of Taoist culture in other places on the growth of the digital economy in a specific city is minimal, therefore, the implementation of *ivDJ* meets the external requirements. The intensity of Taoist culture in each city can be influenced by measurement errors or unobservable factors. Consequently, the relevance condition is satisfied by the use of the *ivDJ* method. The IV approach is employed to re-estimate Equation (1), with *Deco* serving as the dependent variable and *DJ* as the independent variable. The Cragg–Donald Wald F statistic for the weak instrumental variable (IV) test is 2332.232, significantly exceeding the crucial value of 16.38 at a 10 % significance level. Consequently, we can conclude that the instrumental variable, *ivDJ*, successfully passes the weak IV test.

By employing the IV with *ivDJ* as the instrumental variable, Equation (1) is re-estimated. The outcome of this estimation is presented in Column (1) of Panel A in Table 5. Given the potential endogeneity of the control variables, this research employs a lag of one period for all control variables and proceeds to re-evaluate Equation (1) using the instrumental variable (IV) approach. The outcomes of this analysis are then presented in Column (2) of Panel A in Table 5. The findings indicate that the coefficients of Taoist cultural intensity (*DJ*) exhibit a statistically significant positive relationship at a significance level of 1 % or 5 %. Thus, under the assumption of exogeneity, the first hypothesis (H1) remains valid.

**Table 5:** Robustness checks of equation (1).

Panel A				
	(1)	(2)	(3)	(4)
Variables	*Deco*	*Deco*	*fDeco*	*Deco*
				
*DJ*	0.0410***	0.0144**	0.0890***	
	(0.0075)	(0.0058)	(0.0174)	
*rDJ*				0.1036***
				(0.0143)
				
Individual	YES	YES	YES	YES
Province	YES	YES	YES	YES
Control variables	YES	YES	YES	YES
				
Observations	1840	1555	1840	1840
N	229	229	229	229
R^2^	0.7599	0.8850	0.4095	0.7065
Panel B				
	(1)	(2)	(3)	(4)
Variables	*Deco*	*Deco*	*Deco*	*Deco*
				
*rrDJ*	0.0003***		0.0002***	
	(0.0001)		(0.0001)	
*rDJ*		0.2902***		
		(0.0831)		
*DJ*				0.0929***
				(0.0153)
*Ceff*				0.0411***
				(0.0075)
				
Individual	YES	YES	YES	YES
Province	YES	NO	NO	YES
Control variables	YES	YES	YES	YES
Individual (city) effect	NO	YES	YES	NO
				
Observations	1840	1840	1840	1840
N	229	229	229	229
R^2^	0.6638	0.7770	0.7765	0.7065

Note: IV is robust standard error.

#### 4.3.2 Other robustness tests

##### 4.3.2.1 Substituting the dependent variable

By considering *fDeco* as the dependent variable and accounting for time and province fixed effects, we proceed to re-evaluate Equation (1). The outcome of this re-estimation is presented in Column (3) of Panel A in Table 5. The results of the study provide confirmation that the presence of Taoist culture contributes to the progress of the digital economy. This validation supports the stability of the conclusion stated in hypothesis H1.

##### 4.3.2.2 Replacing independent variables

Given the increasing impact of Taoist culture, we proceed to analyze the relationship between *rDJ* (the independent variable) and its influence. To account for the impacts of time and province, we control for these variables and re-evaluate Equation (1). The findings are presented in Column (4) of Panel A in Table 5. The phenomenon of conformity can also exert an influence on individuals' attitudes towards Taoist culture, as it exhibits a close association with the size of social groups. Equation (1) is re-estimated in this analysis, incorporating *rrDJ* as an independent variable, while accounting for the effects of time and population size. Time and provincial fixed effects are controlled for, and the findings are presented in Column (1) of Panel B in Table 5. The findings of this study provide confirmation that the presence of Taoist culture contributes to the advancement of the digital economy. This validation supports the stability of the conclusion stated in Hypothesis 1.

##### 4.3.2.3 Changing the estimation model

The independent variables *rDJ* and *rrDJ* are utilized in the re-estimation of Equation (1) through the incorporation of individual fixed effects. Taking into account the temporal dimension and the psychological concept of conformity, the variables *rDJ* and *rrDJ*, which are independent in nature, exhibit changes over a period of time. Additionally, the city fixed effect can be employed to recalibrate Equation (1). The results presented in columns (2) and (3) of Panel B in Table 5 demonstrate that Taoist culture contributes to the advancement of digital economy growth. This finding further confirms the stability of the conclusion stated in H1.

##### 4.3.2.4 Carbon efficiency control

The enhancement of political accomplishments by city governments necessitates the prioritization of local economic growth. In recent times, the foremost environmental predicament is attributed to the detrimental effects of carbon emissions. The mitigation of carbon emissions is of paramount importance for municipal administrations in order to enhance their political efficacy. The digital economy exhibits a sustained capacity to mitigate emissions over an extended period of time. By adopting this approach, municipal administrations can expedite the advancement of the digital economy and enhance their political accomplishments. This implies that the growth of cities' digital economy might be influenced more by carbon emissions rather than the influence of Taoist culture. The carbon efficiency (*Ceff*) is calculated by dividing the real GDP of the city by the amount of carbon dioxide emissions, as indicated in Equation (1). After accounting for time and provincial fixed effects, the outcome is displayed in Column (4) of Panel B in Table 5. The results, after accounting for carbon efficiency (*Ceff*), suggest that Taoist culture contributes to the progress of the digital economy. This further supports the stability of the conclusion made in hypothesis H1.

## 5 Mechanism tests

Our theoretical analysis demonstrates that Taoist culture promotes digital economy development through financial decentralization and financial technology. We next test the mechanisms of the two channels applying mediating effect analysis.

### 5.1 Financial decentralization channel

In order to reassess Equations (2), (3), (4), we incorporate the level of financial decentralization (*Fd*) in cities as the mediating variable. The outcomes of this analysis are presented in Columns (1)–(3) of Panel A in Table 6. In Panel A, the coefficient of Taoist cultural intensity (*DJ*) in Column (1) is statistically significant at the 1 % level, suggesting the presence of a significant overall effect. The coefficient of Taoist culture intensity (*DJ*) in Column (2) demonstrates statistical significance at the 1 % level of significance. Similarly, the coefficient of the mediating variable of cities' financial decentralization (*Fd*) in Column (3) also exhibits statistical significance at the 1 % level. These findings support the existence of financial decentralization channels, thereby confirming H2. The relationship between Taoist culture intensity (*DJ*) and the degree of financial decentralization in cities (*Fd*) suggests that Taoist culture has the potential to enhance financial decentralization, hence promoting the development of the digital economy.

**Table 6:** Estimation results of financial decentralization channels.

Panel A					
	(1)	(2)	(3)	(4)	(5)
Variables	*Deco*	*Fd*	*Deco*	*Fd*	*Deco*
					
*DJ*	0.1014***	0.0071***	0.0455***	0.0046***	0.0227***
	(0.0158)	(0.0010)	(0.0096)	(0.0007)	(0.0070)
*Fd*			6.5803***		5.4191***
			(1.0407)		(0.8383)
					
Individual	YES	YES	YES	YES	YES
Province	YES	YES	YES	YES	YES
Control variables	YES	YES	YES	YES	YES
					
Observations	1840	1840	1840	1840	1840
N	229	229	229	229	229
R^2^	0.6731	0.7255	0.8466	0.7853	0.8532
Panel B					
	(1)	(2)	(3)	(4)	(5)
Variables	*Deco*	*Fd*	*Deco*	*Fd*	*Deco*
					
*rDJ*	0.1036***	0.0051***	0.0466***	0.0044***	0.0219***
	(0.0143)	(0.0009)	(0.0090)	(0.0007)	(0.0067)
*Fd*			6.5358***		5.4001***
			(1.0400)		(0.8413)
					
Individual	YES	YES	YES	YES	YES
Province	YES	YES	YES	YES	YES
Control variables	YES	YES	YES	YES	YES
					
Observations	1840	1840	1840	1840	1840
N	229	229	229	229	229
R^2^	0.6729	0.7261	0.8460	0.7854	0.8532
Panel C					
	(1)	(2)	(3)	(4)	(5)
Variables	*fDeco*	*Fd*	*fDeco*	*Fd*	*fDeco*
					
*DJ*	0.0890***	0.0071***	0.0319***	0.0046***	0.0218***
	(0.0174)	(0.0010)	(0.0090)	(0.0007)	(0.0063)
*Fd*			8.1161***		8.3279***
			(1.0375)		(0.7407)
					
Individual	YES	YES	YES	YES	YES
Province	YES	YES	YES	YES	YES
Control variables	YES	YES	YES	YES	YES
					
Observations	1840	1840	1840	1840	1840
N	229	229	229	229	229
R^2^	0.6331	0.7255	0.8683	0.7853	0.8719

Note: all instrumental variables pass the validity test.

When estimating Equation (3) with cities' degree of financial decentralization (*Fd*) as the mediating variable, it is challenging to form a two-way causal relationship between financial decentralization and Taoist culture intensity (*DJ*); however, endogeneity problems may still occur due to measurement errors or unobservable factors. Taking *ivDJ* as the IV and cities' financial decentralization level (*Fd*) as the mediating variable, Equation (3) is re-estimated using the IV approach. The results are presented in Column (4) of Panel A in Table 6. In addition, when estimating Equation (4), cities' degree of financial decentralization can affect digital economy development. In addition, enterprises' digital transformation can improve the problem of information asymmetry [33], which strengthens financial institutions' financial risk control. When financial decentralization generates regional financial risks [40], digital economy development will help control the financial risks associated with financial decentralization, encouraging city governments to courageously improve the level of financial decentralization. Therefore, the digital economy may also affect financial decentralization. Thus, there is a two-way causal relationship between digital economy development and cities' degree of financial decentralization, making the level of cities' financial decentralization (*Fd*) endogenous. Referencing Kim et al. (2014) [44] and Chen et al. (2023) [9], taking the mean amount of financial decentralization observed in other cities during the corresponding year as the IV (*ivFd*), together with the IV (*ivDJ*), this study uses the IV method to re-estimate the estimation Equation (4). The results are shown in Column (5) of Panel A in Table 6. It can be seen that, excluding endogeneity, Taoist culture can improve the level of city's financial decentralization, advancing digital economy development; thus, H2 remains valid.

Based on the aforementioned methodology, the independent variable *rDJ* is utilized to re-evaluate Equations (2), (3), (4). The findings are displayed in panel B of Table 6, wherein we substitute the dependent variable with *fDeco*, utilize *DJ* as the independent variable, and subsequently re-evaluate Equations (2), (3), (4). The findings are displayed in Panel C of Table 6. Panels B and C additionally demonstrate the potential of Taoist culture to enhance the financial decentralization of cities, hence promoting the advancement of digital economy development. Thus, the validity of H2 is maintained even after controlling for endogeneity.

### 5.2 Financial technology channel

By considering the level of financial technology (Fintech) in various cities as the mediating variable, we have recalculated Equations (2), (3), (4). The outcomes of this analysis are displayed in Columns (1)–(3) of Panel A in Table 7. The findings provide support for the existence of financial technology channels, hence confirming hypothesis H3. The correlation between the intensity of Taoist culture (*DJ*) and the presence of financial technology (*Fintech*) in city suggests that Taoist culture has the potential to enhance the advancement of digital economy development by improving the level of financial technology.

**Table 7:** Estimated results of financial technology channels.

Panel A					
	(1)	(2)	(3)	(4)	(5)
Variables	*Deco*	*FinTech*	*Deco*	*FinTech*	*Deco*
					
*DJ*	0.1014***	0.0120***	0.0803***	0.0060***	0.0286***
	(0.0158)	(0.0034)	(0.0150)	(0.0020)	(0.0070)
*FinTech*			1.1759***		1.6259***
			(0.1240)		(0.1616)
					
Individual	YES	YES	YES	YES	YES
Province	YES	YES	YES	YES	YES
Control variables	YES	YES	YES	YES	YES
					
Observations	1840	1840	1840	1840	1840
N	229	229	229	229	229
R^2^	0.6731	0.9891	0.7270	0.9909	0.7780
Panel B					
	(1)	(2)	(3)	(4)	(5)
Variables	*Deco*	*FinTech*	*Deco*	*FinTech*	*Deco*
					
*rDJ*	0.1036***	0.0125***	0.0819***	0.0058***	0.0274***
	(0.0143)	(0.0031)	(0.0135)	(0.0019)	(0.0067)
*FinTech*			1.1622***		1.6207***
			(0.1235)		(0.1619)
					
Individual	YES	YES	YES	YES	YES
Province	YES	YES	YES	YES	YES
Control variables	YES	YES	YES	YES	YES
					
Observations	1840	1840	1840	1840	1840
N	229	229	229	229	229
R^2^	0.6729	0.9891	0.7264	0.9909	0.7782
Panel C					
	(1)	(2)	(3)	(4)	(5)
Variables	*fDeco*	*FinTech*	*fDeco*	*FinTech*	*fDeco*
					
*DJ*	0.0890***	0.0120***	0.0843***	0.0060***	0.0425***
	(0.0174)	(0.0034)	(0.0173)	(0.0020)	(0.0084)
*FinTech*			0.2491**		0.9739***
			(0.1208)		(0.1898)
					
Individual	YES	YES	YES	YES	YES
Province	YES	YES	YES	YES	YES
Control variables	YES	YES	YES	YES	YES
					
Observations	1840	1840	1840	1840	1840
N	229	229	229	229	229
R^2^	0.6331	0.9891	0.6477	0.9909	0.7160

When attempting to estimate Equation (3) using the degree of financial technology (*Fintech*) in cities as the mediating variable, establishing a bidirectional causal relationship between cities' financial technology and the intensity of Taoist culture (*DJ*) is also problematic. However, the presence of endogeneity issues may arise due to measurement errors or unobservable factors. In this study, the instrumental variable (IV) used is *ivDJ*, whereas the mediating variable is the degree of financial technology (*Fintech*) in cities. The IV method is employed to re-estimate Equation (3), and the resulting findings are presented in Column (4) of Panel A in Table 7. Furthermore, the estimation of Equation (4) suggests that financial technology has the potential to impact the development of the digital economy. Specifically, the digital economy can play a role in mitigating information asymmetry, particularly in relation to the credit supply and demand dynamics. This, in turn, can lead to a reduction in credit risk for banks and incentivize them to prioritize innovation in financial technology. Consequently, the overall development of financial technology can be fostered. Hence, there exists a bidirectional causal association between the advancement of the digital economy and the level of financial technology within cities, wherein financial technology (*Fintech*) is considered an endogenous factor. The IV technique is utilized in this study, wherein the practice of financial decentralization channels is referenced. Additionally, the mean of other cities' financial technology development in the same year as the instrumental variable (*ivFintech*) is incorporated, along with the instrumental variable (*ivDJ*), to re-estimate Equation (4). The findings are displayed in Column (5) of Panel A of Table 7. The findings in Panel A of Table 7, specifically columns (4) and (5), provide empirical evidence supporting the positive impact of Taoist culture on the degree of financial technology in cities. This, in turn, contributes to the development of the digital economy. These results further validate the hypothesis H3, even after controlling for endogeneity.

equations (2), (3), (4) are re-estimated, and the outcomes are presented in Panels B and C of Tables 7 and in comparison with financial decentralization pathways. The result can be considered valid if endogeneity is not taken into account. The integration of Taoist culture has the potential to enhance the financial technology sector in cities, hence promoting the advancement of digital economy development.

## 6 Discussion

We investigate the impact of Taoist culture on the digital economy based on a sample of 229 Chinese cities, and found that Taoist culture can promote digital economy development. Our conclusions align with those of Chen et al. (2023) [9] and Li (2015) [4]. Chen et al. (2023) found that Taoist culture enhances employees' positive psychological capital toward enterprises, which promotes innovation and benefits digital inclusive finance [9]. Digital economy development also requires enterprises to innovate digital technology and digital transformation approaches, both of which are aspects of enterprise innovation. This indicates that our conclusions are consistent with those of Chen et al. (2023). Li (2015) [4] argued that the imaginative and creative nature of Taoist culture, which encourages novel ideas, has a role similar to Western science fiction thinking, stimulating Chinese creativity and promoting innovation. This means that Taoist culture can advance Chinese employees’ digital technology and digital transformation innovation, promoting digital economy development.

Our research demonstrates that Taoist culture benefits digital economy development by promoting financial technology innovation. This conclusion is also consistent with Chen et al. (2022) [22], who determined that financial technology promotes digital economy development based on a provincial sample [22]. We also reveal that financial technology promotes digital economy development by conducting mechanism tests based on city samples; however, our research also uncovers inconsistencies with Chen et al. (2022) [22]. Chen et al. (2022) found that financial decentralization advanced by provincial governments does not advance digital economy development [22]. Our research reveals that financial decentralization from city governments benefits the digital economy development. The rationale for this may be that provincial governments' allocation of financial resources is significantly higher than city governments’ allocation of financial resources, resulting in an excessively negative impact on digital economy development.

## 7 Conclusion

Based on basic concepts of Taoist culture, this study empirically investigates its impact on digital economy development and its mechanisms. Previous research has explored the influencing factors of digital economy development from dimensions of technology [19], finance [22], legal systems, and markets [20,21]; however, limited studies have examined influences on the digital economy from a cultural perspective. Our research endeavors to contribute in this regard. Previous studies have explored the impact of Taoist culture from both macro [9,10]and micro [[11], [12], [13]] perspectives, but have not yet expanded the scope of this research to the digital economy. Our research examines this consideration.

This study has some theoretical and practical significance. **First, policymakers and business managers should moderately delegate power**. Our analysis demonstrates that the inaction ideology of Taoist culture can inspire policymakers and business managers to govern collaboratively, not act recklessly, act accordingly, and courageously delegate power, which encourages lower local governments and enterprise employees to actively innovate and promote digital economy development. This indicates that policymakers could actively formulate principled regulations when developing policies so that enterprises will implement these principled regulations, leaving space for moderately delegating power for enterprises to exert enthusiastic innovation efforts. Enterprise managers can also develop principled regulations to be implemented by employees, leaving space for employees to unleash their talent and creativity and decentralizing power appropriately.

**Second, policymakers and business managers should maintain strategic focus and face innovation in the digital economy calmly**. Our research shows that quietness is one of the fundamental concepts of Taoist culture, which pursues spiritual unity and facilitates calmness, thereby encouraging lower local governments and enterprise employees to focus on innovation, which promotes digital economy development. Digital economy development requires active and ongoing digital innovation, which can improve social welfare, while also having negative impacts (such as privacy breaches). Faced with negative impacts, policymakers must remain calm and respond cautiously, and avoid rejecting innovation in a one-size-fits-all manner. Similarly, business managers must also remain calm and carefully examine the mechanism of avoiding negative impacts, rather than directly denying innovation.

We examine the impact and mechanisms of Taoist culture on the digital economy. Many influencing factors affect digital economy development, with digital technology at its core. How Taoist culture affects digital technology innovation and digital economy development is not examined in this study; a deficiency that also presents a potential future research direction. In addition, other pathways may affect the impact of Taoist culture on digital economy development, which can also be investigated in the future.

## Data availability

Data and code are available by email to the correspondence author.

Xing Wu: Analyzed and interpreted the data; Contributed reagents, materials, analysis tools or data; Wrote the paper.

## Declaration of interest's statement

The authors declare no conflict of interest.

## CRediT authorship contribution statement

**Xiaohui Chen:** Writing - original draft, Methodology, Formal analysis, Data curation, Conceptualization. **Xing Wu:** Writing - review & editing, Supervision, Software, Funding acquisition, Formal analysis.

## Declaration of competing interest

The authors declare that they have no known competing financial interests or personal relationships that could have appeared to influence the work reported in this paper.
